# Correlation of Blood Glucose and Pancreatic Islet Function with Serum Retinol-Binding Protein 4, Serum Cystatin C, and Human New Satiety Molecule Protein-1 in Pregnant Women with Gestational Diabetes Mellitus

**DOI:** 10.1155/2022/4247412

**Published:** 2022-07-09

**Authors:** Haiyan Zhang, Tianhong Sun

**Affiliations:** Dongying District Maternal and Child Health Hospital, Department of Gynaecology and Obstetrics, Dongying, Shandong, China

## Abstract

**Objective:**

To investigate the correlation of blood glucose and islet function with serum retinol-binding protein 4, serum cystatin C, and nesfatin-1 levels in women with gestational diabetes mellitus.

**Methods:**

Between June 2018 and June 2020, 70 patients with gestational diabetes mellitus were included in a study group and 70 healthy pregnant women were recruited into a healthy group. Alterations in fasting blood glucose (FPG), glycated hemoglobin (HbA1c), fasting serum insulin (FINS), homeostatic model assessment for insulin resistance (HOMA-IR), serum retinol-binding protein 4 (RBP4), serum cystatin C (CysC), and nesfatin-1 of all eligible participants were analyzed, and the occurrence of complications was recorded. Correlation analysis of serum RBP4, serum CysC, and nesfatin-1 levels with blood glucose and islet function in women with gestational diabetes mellitus was performed.

**Results:**

Gestational diabetes mellitus was associated with significantly higher levels of FPG, HbA1c, and HOMA-IR and lower levels of FINS (6.58 ± 1.41, 9.24 ± 1.09, 3.21 ± 2.03, 8.23 ± 2.21) versus a healthy condition (5.23 ± 0.85, 7.61 ± 0.67, 2.42 ± 1.14, 10.54 ± 2.15) (*P* < 0.05). Women with gestational diabetes mellitus showed significantly higher levels of serum RBP4, serum CysC, and nesfatin-1 (62.45 ± 7.86, 1.95 ± 0.59, 2.65 ± 0.49) versus healthy pregnant women (45.48 ± 6.15, 1.03 ± 0.67, 1.42 ± 0.62) (*P* < 0.05). With serum RBP4, serum CysC, and nesfatin-1 as dependent variables, univariate correlation analysis showed that serum RBP4, serum CysC, and nesfatin-1 levels were positively correlated with FPG and HbA1c levels and HOMA-IR, and negatively correlated with FINS in women with gestational diabetes mellitus (*P* < 0.05). Gestational diabetes mellitus resulted in a significantly higher incidence of preterm delivery, cesarean section, excess amniotic fluid, and premature rupture of membranes versus a healthy status (*P* < 0.05).

**Conclusion:**

Glucose metabolism and islet function in women with gestational diabetes are significantly correlated with serum RBP4, serum CysC, and nesfatin-1 levels, which shows great potential for the prevention and treatment of gestational diabetes mellitus and perinatal complications.

## 1. Introduction

Gestational diabetes mellitus (GDM) [1] refers to diabetes mellitus that only develops during pregnancy with confirmed normal glucose metabolism or potentially reduced glucose tolerance before pregnancy [2, 3], as per the diagnostic criteria for gestational diabetes issued by the Ministry of Health of the People's Republic of China on July 1, 2011 [4]. Due to genetic and environmental factors and dietary changes [5, 6], the current incidence of GDM in China exceeds 10% with an escalating trend annually, which is similar to the pathogenesis of type 2 diabetes mellitus (T2DM). Hyperglycemia in pregnancy may lead to abnormal fetal development with an incidence of miscarriage of 15%–30%, posing a considerable risk to pregnancy, delivery, maternal long-term prognosis, and perinatal infants [7]. The etiology of GDM has not been fully elucidated, and its development may be associated with increased maternal and placental secretion of anti-insulin hormones [8], which can result in intrauterine distress, hypoglycemia, giant fetuses, obesity in the offspring, diminished long-term cognitive ability, and increased risk of T2DM, and even an increased incidence of adverse outcomes such as postpartum metabolic disorders, hyperhydramnios, obstructed shoulder labor, and preterm delivery in pregnant women [9, 10]. It has been reported that abnormal levels of serum retinol-binding protein 4 (RBP4) [11], serum cystatin C (CysC), and nesfatin-1 are directly related to insulin resistance in women with gestational diabetes mellitus. RBP4 is a novel adipocytokine [12] whose abnormal expression correlates with insulin resistance [13]. Serum CysC is involved in the dynamic balance of production and degradation of the vascular wall and extracellular matrix [8, 14]. Nesfatin-1 is a secretory peptide that may function in the regulation of blood glucose levels in diabetes mellitus. Accordingly, this study was conducted to investigate the correlation of blood glucose and islet function with serum retinol-binding protein 4, serum cystatin C, and nesfatin-1 levels in women with gestational diabetes mellitus so as to provide a basis for clinical diagnosis and a laboratory reference for monitoring and treatment of the disease.

## 2. Materials and Methods

### 2.1. Baseline Data

Between June 2018 and June 2020, 70 patients with gestational diabetes mellitus were included in a study group and 70 healthy pregnant women were recruited in a healthy group. The clinical features of the study group (aged 23–35 years, mean age of 25.68 ± 4.27 years, gestational weeks of 35–40 weeks, mean gestational weeks of 35.01 ± 2.21 weeks, gravidity of 1–3 times, mean gravidity of 2.28 ± 0.61 times) were comparable with those of the healthy group (aged 22–36 years, mean age of 27.02 ± 3.54 years, gestational weeks of 33–41 weeks, mean gestational weeks of 35.37 ± 1.99 weeks, gravidity of 1–3 times, mean gravidity of 2.36 ± 0.57 times).

### 2.2. Inclusion and Exclusion Criteria

Inclusion criteria: patients who met the diagnostic criteria related to GDM in the Guidelines for the Diagnosis and Treatment of Gestational Combined Diabetes Mellitus (2014) developed by the Obstetrics and Gynecology Section of the Chinese Medical Association, without prior use of hypoglycemic drugs, and who provided written informed consent were included.

Exclusion criteria: patients with hypertension, chronic nephritis, and coronary artery disease, with multiple pregnancies, or a history of psychiatric disorders were excluded.

### 2.3. Methods

All pregnant women fasted from the night before blood sample collection. 5 ml of fasting venous blood was collected in the early morning of the next day and centrifuged at 3000 r/min for 10 min, and the supernatant was collected without anticoagulation and then stored at −70°. Fasting blood glucose (FPG) level was determined by the glucose oxidase method, glycated hemoglobin (HbA1c) level was determined by the high-pressure liquid phase method, fasting serum insulin (FINS) was determined by radioimmunoassay, and homeostatic model assessment for insulin resistance (HOMA-IR) was evaluated by the latest improved HOMA model. Serum RBP4 (kit purchased from R&D System, USA) and nesfatin-1 (kit purchased from PHOENIX, USA) levels were determined by ELISA, and serum CysC levels (kit purchased from Shanghai Kehua Biological Engineering Co., Ltd.) were determined by the turbidimetric assay. The instruments included a LAB systems Muhiskan MK3 enzyme marker and a Beckman fully automated biochemical analyzer. All assays were performed in strict accordance with the operating instructions.

### 2.4. Outcome Measures

1. Glucose and islet function: FPG, HbA1c, FINS levels, and HOMA-IR index were recorded and compared between the two groups of pregnant women. HOMA-IR=FBG×FINS/22.5.
2. Serum RBP4, serum CysC, and nesfatin-1 levels were monitored and recorded in the two groups of pregnant women.
3. Correlation: the correlation of serum RBP4, serum CysC, and nesfatin-1 levels with FPG, HbAlc, FINS, and HOMA-IR index in women with gestational diabetes was analyzed and compared.
4. Complications: the occurrence of perinatal complications (excess amniotic fluid, premature rupture of membranes, preterm delivery, cesarean section, and postpartum hemorrhage) in the two groups of pregnant women was recorded and compared. The investigators and analysts counted the number of perinatal complications and used it to divide the total number to obtain the incidence of complications.

### 2.5. Statistical Analysis

SPSS 22.0 was used for data analyses. The measurement data were expressed as ($\bar{\text{x}}$ ± *s*) and processed using the *t*-test. The count data were expressed as the number of cases (rate) and analyzed using the chi-square test. Pearson correlation analysis was used for the correlation analysis of the data. Differences were considered statistically significant at *P* < 0.05.

## 3. Results

### 3.1. Baseline Data

The two groups presented similar baseline data (*P* > 0.05).

### 3.2. Blood Glucose and Islet Function

Gestational diabetes mellitus was associated with significantly higher levels of FPG, HbA1c, and HOMA-IR and lower levels of FINS (6.58 ± 1.41, 9.24 ± 1.09, 3.21 ± 2.03, 8.23 ± 2.21) versus a healthy condition (5.23 ± 0.85, 7.61 ± 0.67, 2.42 ± 1.14, 10.54 ± 2.15) (*P* < 0.05) (Table 1).

### 3.3. Serum RBP4, Serum CysC, and Nesfatin-1

Women with gestational diabetes mellitus showed significantly higher levels of serum RBP4, serum CysC, and nesfatin-1 (62.45 ± 7.86, 1.95 ± 0.59, 2.65 ± 0.49) versus healthy pregnant women (45.48 ± 6.15, 1.03 ± 0.67, 1.42 ± 0.62) (*P* < 0.05) (Table 2).

### 3.4. Correlation

With serum RBP4, serum CysC, and nesfatin-1 as dependent variables, univariate correlation analysis showed that serum RBP4, serum CysC, and nesfatin-1 levels were positively correlated with FPG and HbA1c levels and HOMA-IR, and negatively correlated with FINS in women with gestational diabetes mellitus (*P* < 0.05) (Table 3).

### 3.5. Complication

There were 9 (12.86%) cases of preterm delivery, 36 (51.43%) cases of cesarean delivery, 11 (15.71%) cases of excessive amniotic fluid, 4 (5.71%) cases of premature rupture of membranes, and 4 (5.71%) cases of postpartum hemorrhage among the eligible patients, and 2 (2.86%) cases of preterm delivery, 15 (21.43%) cases of cesarean delivery, 2 (2.86%) cases of excessive amniotic fluid, and 2 (2.86%) cases of postpartum hemorrhage among healthy pregnant women. Gestational diabetes mellitus was associated with a significantly higher incidence of preterm delivery, cesarean section, excess amniotic fluid, and premature rupture of membranes versus a healthy status (*P* < 0.05) (Table 4).

## 4. Discussion

The current prevalence of gestational diabetes mellitus (GDM) exceeds 10%, which poses a great threat to the health of pregnant women and fetuses [15]. Gestational diabetes mellitus is mainly staged based on the age at which the patient developed diabetes, the duration of the disease, and the presence of vascular complications (White classification) to determine the severity and prognosis of the disease [16]. Abnormal glucose metabolism during pregnancy has been reported [17] to be associated with adverse maternal outcomes, such as abnormal maternal amniotic fluid, premature rupture of membranes, giant babies, or intrauterine distress, with varying degrees of renal impairment, which mostly requires lipid management [5] to facilitate the recovery of their glomerular filtration function. It has been found that the development of gestational diabetes is closely related to the levels of several cytokines, and insulin resistance in women with GDM showed a direct association with serum RBP4, serum CysC, and nesfatin-1 levels, which may potentially contribute to the diagnosis and prevention of GDM. Serum RBP4 is a novel adipocytokine and a secreted retinol-binding protein that transports retinol through the hepatic circulation [18, 19]. With the decline of glomerular filtration function and renal blood flow, RBP4 will accumulate in various forms and increase the blood RBP4 concentration. Serum CysC is involved in the dynamic balance of vascular wall and extracellular matrix production and degradation [14]. CysC is a cysteine proteinase inhibitor produced by most nucleated cells and has been considered a replacement for serum creatinine or even an alternative endogenous marker for glomerular filtration rate (GFR). The plasma concentration of CysC is stable, since it can be freely filtered through the glomerular membrane and reabsorbed and catabolized by renal tubular cells. Nesfatin-1 is a novel secretory peptide secreted by the brainstem and hypothalamus and was found by Stengel et al. to increase the rate of fat conversion in humans to control body fat content.

The results of the present study showed that gestational diabetes mellitus was associated with significantly higher levels of FPG, HbA1c, and HOMA-IR and lower levels of FINS versus a healthy condition (*P* < 0.05), which is attributed to the inability of the body function of pregnant women with restricted insulin secretion to compensate for the increased insulin demand, which results in abnormal FPG, HbA1c levels, and HOMA-IR index. This result is consistent with the findings of Xie and Guan et al. Previous studies have demonstrated that abnormal glucolipid metabolism in women with GDM is closely related to abnormal blood glucose levels and islet function, mainly due to the insufficiency of islet function in women with GDM to improve insulin resistance during pregnancy. Here, women with gestational diabetes mellitus showed significantly higher levels of serum RBP4, serum CysC, and nesfatin-1 versus healthy pregnant women (*P* < 0.05), indicating a possible association of abnormal serum RBP4, serum CysC, and nesfatin-1 levels with disease progression. Moreover, univariate correlation analysis in the present study showed that serum RBP4, serum CysC, and nesfatin-1 levels were positively correlated with FPG and HbA1c levels and HOMA-IR, and negatively correlated with FINS in women with gestational diabetes mellitus (*P* < 0.05). Abnormally elevated levels of serum RBP4, serum CysC, and nesfatin-1 may lead to abnormal glucose metabolism and enhanced insulin resistance in pregnant women, which consequently aggravates GDM. The aberrant release of RBP4 is associated with altered pancreatic islet function, and ameliorated serum RBP4 levels can enhance insulin sensitivity and maintain glucose stability. Serum CysC is a good endogenous marker that reflects the glomerular filtration rate [20], and nesfatin-1 promotes fat consumption in the body and contributes to the reduction of blood glucose levels, so abnormal glucose metabolism and insulin resistance in women with gestational diabetes may be jointly determined by multiple factors. It has been found that abnormalities in serum RBP4, serum CysC, and nesfatin-1 in women with GDM may result in multiple complications and pose a great threat to maternal and infant health. The results of the present study demonstrated that gestational diabetes mellitus was associated with a significantly higher incidence of preterm delivery, cesarean section, excess amniotic fluid, and premature rupture of membranes versus a healthy status, indicating the significance of the analysis and monitoring of serum RBP4, serum CysC, and nesfatin-1 levels to prevent and manage complications in women with GDM, which is similar to the research results by Xu et al. Additionally, traditional Chinese medicine believes that the pathogenesis of gestational diabetes mellitus is derived from deficiency of kidney essence and spleen, and is characterized by abnormal metabolism of qi, blood, and body fluids. It is also closely related to liver fire, phlegm-dampness, and blood stasis. The treatment is mainly based on the principle of “replenishing the deficiency, purging the excess and treating the symptoms.” The treatment focuses on nourishing the kidney and the yin, strengthening the spleen, and nourishing the qi to treat the root cause. Moreover, soothing the liver, removing dampness, clearing heat, and promoting blood circulation are key methods to alleviate the symptoms.

The small sample size is a major limitation of this study. Yet, this study is a pilot clinical study, so a minimum sample size was used to investigate our hypothesis.

In conclusion, glucose metabolism and islet function in women with gestational diabetes are significantly correlated with serum RBP4, serum CysC, and nesfatin-1 levels, which shows great potential for the prevention and treatment of gestational diabetes mellitus and perinatal complications in pregnant women.

## Figures and Tables

**Table 1:** Comparison of blood glucose and islet function ($\bar{x}$ ± *s*).

Groups	*N*	FPG (mmol/L)	HbA1c (%)	FINS (mU/L)	HOMA-IR index
Study group	70	6.58 ± 1.41	9.24 ± 1.09	8.23 ± 2.21	3.21 ± 2.03
Healthy group	70	5.23 ± 0.85	7.61 ± 0.67	10.54 ± 2.15	2.42 ± 1.14
*T*	—	6.860	10.659	6.268	2.839
*P* value	—	<0.001	<0.001	<0.001	0.005

FPG, fasting blood glucose; HbA1c, glycated hemoglobin; FINS, fasting serum insulin, HOMA-IR, homeostatic model assessment for insulin resistance.

**Table 2:** Comparison of blood glucose and islet function ($\bar{x}$ ± *s*).

Groups	*n*	Serum RBP4 (mg/L)	Serum CysC (mg/L)	Nesfatin-1 (*μ*g/L)
Study group	70	62.45 ± 7.86	1.95 ± 0.59	2.65 ± 0.49
Healthy group	70	45.48 ± 6.15	1.03 ± 0.67	1.42 ± 0.62
*T*	—	14.226	8.622	13.022
*P* value	—	<0.001	<0.001	<0.001

RBP4, serum retinol-binding protein 4; CysC, serum cystatin C.

**Table 3:** Correlation analysis.

Variables	Serum RBP4		Serum CysC		Nesfatin-1	
	*r*	*P* value	*r*	*P* value	*r*	*P* value
FPG	0.411	0.001	0.287	0.029	0.378	0.003
HbA1c	0.352	0.005	0.298	0.031	0.402	0.001
FINS	−0.351	0.002	−0.301	0.023	−0.411	0.002
HOMA-IR index	0.315	0.012	0.296	0.039	0.325	0.011

FPG, fasting blood glucose; HbA1c, glycated hemoglobin; FINS, fasting serum insulin; HOMA-IR, homeostatic model assessment for insulin resistance; RBP4, serum retinol-binding protein 4; CysC, serum cystatin C.

**Table 4:** Comparison of complications (%).

Groups	*n*	Preterm delivery	Cesarean delivery	Excessive amniotic fluid	Premature rupture of membranes	Postpartum hemorrhage
Study group	70	9 (12.86)	36 (51.43)	11 (15.71)	4 (5.71)	4 (5.71)
Healthy group	70	2 (2.86)	15 (21.43)	2 (2.86)	0 (0.00)	2 (2.86)
*x* ^2^	—	4.834	13.602	6.869	4.118	0.679
*P* value	—	0.028	<0.001	0.009	0.042	0.404

## Data Availability

No data were used to support this study.
